The article "Commentary: One mechanism of Sishen Pill on diarrhea with kidney Yang deficiency syndrome: influencing metabolic function by intestinal microorganisms and enzyme activity mediates the gut-kidney axis" was retracted in 2026. Reasons: compromised peer review; a conflict of interest.

# Commentary: One mechanism of Sishen Pill on diarrhea with kidney Yang deficiency syndrome: influencing metabolic function by intestinal microorganisms and enzyme activity mediates the gut-kidney axis

**DOI:** 10.3389/fcimb.2025.1690941

**Published:** 2025-09-15

**Authors:** Junren Yao, Jiang Lin, Yichuan Xv

**Affiliations:** Department of Gastroenterology, Longhua Hospital, Shanghai University of Traditional Chinese Medicine, Shanghai, China

**Keywords:** Sishen Pill, diarrhea, kidney-Yang deficiency syndrome, gut microbiota, gut-kidney axis

## Introduction

Diarrhea is characterized by increased stool frequency and loose or watery consistency, which in traditional Chinese medicine (TCM) is often attributed to spleen deficiency and accumulation of internal dampness (Ma et al., 2023). Chronic diarrhea may impair spleen Yang, leading to failure of kidney Yang to warm the spleen, ultimately resulting in diarrhea associated with kidney-Yang deficiency syndrome (KYDS). Studies have shown that diarrhea with KYDS significantly presents with intestinal microorganisms dysbiosis, altered digestive enzyme activity, and inflammatory responses in mice (Guo et al., 2024a; Zhou et al., 2023). Additionally, KYDS is associated with disruptions in energy metabolism, including reduced activity of Na^+^/K^+^-ATPase and Ca2^+^-ATPase in various organs and muscles (Chen et al., 2022). Sishen Pill (SSP) is a classic TCM formula widely used for treating diarrhea with KYDS, functioning to warm the kidney and spleen, astringe the intestines, and arrest diarrhea. In modern terms, these concepts correspond to improving systemic energy metabolism and enhancing gastrointestinal digestive function. Modern researches have partly revealed the pharmacological mechanism of SSP such as alleviating mucosal inflammation of intestine, modulating gut microecology, and improving energy metabolism (Chen et al., 2020; Zhu et al., 2023). Therefore, a comprehensive exploration of the effects of SSP on the gut microbiota, enzyme activity, and organ function will help clarify the biological basis of prescription-symptom correspondence between KYDS diarrhea and SSP. Furthermore, analyzing the gut microbiota changes and the effects of SSP intervention in animal models of KYDS diarrhea will help elucidate the microbial-mediated gut-kidney axis.

## General comments

A recent study entitled “One mechanism of Sishen Pill on diarrhea with kidney Yang deficiency syndrome: influencing metabolic function by intestinal microorganisms and enzyme activity mediates the gut-kidney axis” was published in *Frontiers in Cellular and Infection Microbiology* (Zhou et al., 2025). The authors explored the therapeutic effects and mechanisms of SSP using a murine model of diarrhea with KYDS established by adenine and *Folium sennae* co-administration. The study emphasized the role of SSP in reducing harmful gut bacteria, modulating specific enzyme activities, enhancing microbial activity, and mitigating renal oxidative damage. After SSP treatment, the researchers evaluated cultivable microbial colonies, enzyme activity, and metabolic and oxidative stress markers. The results suggested that SSP alleviates diarrhea with KYDS primarily by reducing uric acid levels and *Escherichia coli* (*E. coli*) counts, modulating amylase, sucrase, and protease activities, and increasing spleen and thymus indices along with total bacterial count. The authors concluded that SSP’s regulatory effects on organ indices and oxidative stress may be linked to a microbial–enzymatic regulatory cascade.

Grounded in contemporary microbial ecology theory, the study succinctly but accurately summarized the effect of SSP on KYDS diarrhea and mechanistic effect. First, this study innovatively bridged TCM theory and modern science by linking the TCM pathogenesis of KYDS diarrhea to gut microbiota dysbiosis and gut-kidney axis thereby providing a scientific rationale for the application of classic formulas. Second, a comprehensive evaluation was performed using a multimodal approach that integrated microbial culture, enzyme activity assays, biochemical indicators, and histological analyses. This strategy offered systematic insights into the regulatory role of SSP along the “intestinal-microbiome-enzymatic-organ” axis. Additionally, correlation analyses between serum uric acid levels and gut microbiota suggested that SSP may modulate the microbiota mediated gut-kidney axis, laying a potential foundation for future translational applications.

However, several limitations should be noted. First, the model evaluation criteria could be further improved. Although adenine and *Folium sennae* were used to establish the KYDS diarrhea model, the assessment relied on subjective measures such as diarrhea index and behavioral observations. These methods, to some extent, are less persuasive in confirming model success. Emerging evidence reveals that Yang deficiency is closely associated to dysregulated energy metabolism (Chen et al., 2018; Sun et al., 2023). As key intracellular signaling molecules, cyclic adenosine monophosphate (cAMP) and cyclic guanosine monophosphate (cGMP) participate in cellular regulation and energy metabolism via G-protein-coupled receptors (Kong et al., 2022). cAMP and cGMP levels and their ratio have been established as reliable biomarkers for KYDS animal models (Liu et al., 2020; Chang and Wang, 2025). Specifically, KYDS is associated with decreased cAMP, increased cGMP, and a reduced cAMP/cGMP ratio. Future studies should employ ELISA to quantify serum cAMP and cGMP in model mice, enabling a more objective and refined model evaluation.

Second, the study remained insufficiently comprehensive. Although it enumerated *E. coli*, *Lactobacillus*, and *Bifidobacterium* using microbial culture techniques, these methods were limited in scope and significantly constrained the exploration of SSP’s regulatory role on the microbiota diversity. Further research should employ 16S rRNA sequencing and metagenomic sequencing to assess overall microbial community structural shifts and find the crucial taxa under SSP intervention (Ma et al., 2024). In addition, while superoxide dismutase (SOD) was measured as an indicator of renal oxidative stress response, it is inadequate to explain the SSP-mediated amelioration of renal functional injury and this metric alone does not clarify how SSP modulates oxidative signaling or confers organ protection. NF-κB and Nrf2-Keap pathways are central upstream cascades regulating oxidative stress and inflammation (Jomova et al., 2023). A thorough investigation into these signaling pathways may facilitate the illustration of the mechanistic basis of SSP’s effects. Assessing renal inflammatory cytokines would provide a more comprehensive evaluation of SSP’s protective effects besides oxidative stress.

Finally, the causal chain and rigor underlying SSP’s therapeutic mechanism require strengthening. The causal relationship between gut microbiota and uric acid level cannot be demonstrated based on correlation analysis. Gut microbiota can secrete uricase, degrading uric acid into nitrogen or carbon dioxide, and can also modulate uric acid transporter expression to affect excretion (Zhang et al., 2022; Song et al., 2025). Key transporters include absorptive types such as GLUT9, which reabsorb uric acid, and secretory types such as ABCG2, which promote excretion (Gao et al., 2022). Subsequent studies should quantify uricase activity and levels of uric acid transporters after SSP intervention to better elucidate microbiological role in gut-kidney axis. Moreover, the measured enzyme activity originated from host or microbiota remains unclear, undermining the precision of mechanistic interpretation. The adenine and *Folium sennae* model has been shown to impair the intestinal barrier, reducing occludin and ZO-1 expression while upregulating markers such as D-lactate and diamine oxidase (Zhou et al., 2022; Li et al., 2025). Intestinal proteases may be originated from host cells when mucosal barrier is compromised, while pathogenic microbiota expansion can also release proteases (Pompili et al., 2021). Increased protease activity following SSP treatment could stem either from direct host regulation, such as upregulation of brush border enzyme expression, or from commensal bacteria following suppression of pathogens. Distinguishing host-derived from microbiota-derived enzymes is essential for clarifying SSP’s mechanism and guiding clinical translation. Although the authors have made efforts in this aspect by measuring enzyme activities in mucosa and intestinal contents separately, the future use of germ-free models or rigorous microbiota depletion experiments, such as broad-spectrum antibiotic pretreatment, could help determine the proportion of enzyme activity attributable to microbiota and establish causality between microbiota changes and uric acid levels.

## Discussion

We commend Zhou et al. for their valuable investigation into the mechanisms of SSP in treating diarrhea with KYDS. Their proposed microbiome-enzymatic-gut-kidney axis offers novel insights and potential therapeutic targets for modernizing traditional formulas. However, methodological and experimental refinements are needed to enhance the study’s rigor and scientific validity. Although the results suggest that SSP improves kidney dysfunction by modulating gut microbiota and enzyme activity, higher-quality systematic evaluations are required to establish causality. To definitively separate host and microbiota derived enzymatic contributions, germ-free models or broad-spectrum antibiotic pretreatment can be incorporated into the experimental design to quantify the microbial contribution to enzyme activity. Bacterial depletion efficacy could be verified via 16S rRNA gene-targeted quantitative PCR, while the application of high-throughput sequencing could provide a comprehensive view of SSP’s impact on gut microbiota. On the basis of rigorous microbiota-depletion experiments, subsequent fecal microbiota transplantation (using microbiota from SSP-treated donors) or mono-colonization with either *E. coli* or *Lactobacillus* will be employed to dissect the causal relationship between the gut microbiota and serum uric acid levels.

Previous researches have demonstrated that SSP effectively improves KYDS diarrhea by regulating the disrupted intestinal mucosal microbiota, reducing the accumulation of harmful metabolites, downregulating the expression of inflammatory factors and fortifying the intestinal mucosal barrier (Guo et al., 2024b; Di et al., 2025). The findings from Zhou et al., coupled with existing evidence, suggest that SSP holds significant potential for clinical translation in the management of chronic diarrhea associated with KYDS. Clinically, the ability of SSP to restore gut microbial balance could also benefit patients with functional gastrointestinal disorders, such as irritable bowel syndrome. Overall, SSP demonstrates multi-target therapeutic potential for KYDS diarrhea, but deeper mechanistic studies and research on the safety of clinical applications will facilitate its clinical translation and the modernization of TCM formulas.
